# Analysis of the Impact of Livestock Structure on Carbon Emissions of Animal Husbandry: A Sustainable Way to Improving Public Health and Green Environment

**DOI:** 10.3389/fpubh.2022.835210

**Published:** 2022-02-11

**Authors:** Rubiao Shi, Muhammad Irfan, Guangliang Liu, Xiaodong Yang, Xufeng Su

**Affiliations:** ^1^School of Marxism, Xinjiang University, Urumqi, China; ^2^Department of Public Instruction, Shandong College of Traditional Chinese Medicine, Yantai, China; ^3^School of Management and Economics, Beijing Institute of Technology, Beijing, China; ^4^Center for Energy and Environmental Policy Research, Beijing Institute of Technology, Beijing, China; ^5^Department of Business Administration, Ilma University, Karachi, Pakistan; ^6^School of Economics and Management, Xinjiang University, Urumqi, China; ^7^Center for Innovation Management Research of Xinjiang, Xinjiang University, Urumqi, China; ^8^School of Economics and Management, Tarim University, Alar, China

**Keywords:** livestock structure, animal husbandry, livestock breeding, carbon emission, geographical heterogeneity

## Abstract

Carbon emissions of animal husbandry have been gaining increasing attention due to their high share in global carbon emissions. In this regard, it is essential to assess the regional differences, dynamic evolution patterns, convergence characteristics, and the impact of livestock structure on carbon emissions of animal husbandry. Using data from 30 provincial administrative regions from 2000 to 2018 in China, this study employs the Thiel index method, kernel density analysis, and convergence analysis to quantify the impact of livestock structure on carbon emissions of animal husbandry. The statistical results reveal that carbon emissions of animal husbandry exhibit a rising and declining trend. Specifically, the carbon emissions of animal husbandry are highest in agricultural areas (with a declining trend), followed by agro-pastoral areas (with a declining trend), and the pastoral areas (with a rising trend). It is further revealed that there are no δ convergence and β convergence of carbon emissions of animal husbandry. Finally, essential and useful policy recommendations are put forward to inhibit carbon emissions of animal husbandry.

## Introduction

Carbon emissions from animal husbandry have been emerged as an essential issue, affecting the sustainable development of animal husbandry. Besides, they also have a key constraint to green and low-carbon economic development (1, 2). Excessive carbon emissions exacerbate global warming and deteriorating environmental quality (3–5), obligating humans to face severe risks, such as economic stagnation, health damage, resource shortages, and extreme weather events (6–10). According to the Food and Agriculture Organization of the United Nations (FAO), animal husbandry has contributed to 9% of anthropogenic carbon emissions while emitting 37% of anthropogenic methane, 65% of anthropogenic nitrous oxide, and 64% of anthropogenic nitrogen (11)^1^.

China, the world's largest meat market, consumes 46% of the world's pork, 11% of beef, 18% of chicken, and 48% of lamb (12). However, China's per capita meat consumption is still low compared to that of developed countries. To improve people's living standards, the Chinese government has poured many resources to boost animal husbandry (13). Along with the rising per capita income, China's demand for meat products continues to grow. Among them, beef consumption increased from 5 million tons in 2000 to 7.7 million tons in 2019 (12, 14, 15) (see Figure 1). For example, Figure 1 shows that pork consumption (~20%) accounts for the bulk of meat consumption in terms of livestock structure, while beef (~2%) and mutton (~1%) consumption account for a relatively small share of meat consumption. As for the lamb, China is also the world's largest importer of lamb, with an expected import volume of 1.38 million tons in 2021 (Organisation for Economic Co-operation and Development)^2^. China is also the world's largest producer of livestock products (16). Although the increase in livestock products does improve people's standard of living, the production of livestock products brings a large amount of greenhouse gas emissions such as CH_4_, N_2_O, and CO_2_.

**Figure 1:** Trends of per capita meat consumption (unit: kg) in China. China statistical yearbook.

Therefore, as the world's largest producer of animal husbandry, mitigating carbon emissions of animal husbandry has become an essential scientific issue for China to align with coordinated economic and environmental development and cope with global climate change (16). Similarly, the dual pressure of increasing animal husbandry products and reducing carbon emissions helps improve the efficiency of animal husbandry development and facilitates the high quality of animal husbandry. On the other hand, reducing carbon emissions of animal husbandry is conducive to driving greenhouse gas emissions reduction (17, 18). For instance, Yao et al. (17) use the life cycle assessment method to reveal the evolutionary characteristics of carbon emissions of animal husbandry in China at both temporal and spatial levels, aiming to provide a better perspective for implementing energy conservation and emission reduction at the animal husbandry level. The Chinese government has also been making significant efforts to reduce carbon emissions, mainly the dual carbon target proposed in 2020, which sets new requirements for carbon emission reduction (19)^3^. However, scholars pay more attention to the micro aspects of animal husbandry carbon emissions. For instance, Zhuang and Li (1) study different feeding methods or species' carbon footprints. These micro studies are helpful for people to scientifically understand the carbon emissions of animal husbandry, but they cannot provide a direct reference for the formulation of scientific macro carbon emissions reduction policies of animal husbandry. In addition, some scholars employ the emissions factor method or life cycle method to quantify the carbon emissions of animal husbandry at the macro level, followed by descriptive statistics to analyze the regional differences. However, the above-mentioned studies only explain the significant differences in carbon emissions from animal husbandry among various areas. Still, the trends and sources of the differences have rarely been discussed. Therefore, studying the characteristics and drivers of carbon emissions in animal husbandry is not only conducive to providing important policy references for exploring the path of carbon emissions reduction, but also beneficial to achieving low-carbon development in animal husbandry. Meanwhile, it can also provide some implications for other developing countries with similar development to China in the formulation of carbon emissions reduction policies (20, 21).

To sum up, this study may enrich the existing research in the following dimensions. *Firstly*, to examine the temporal and spatial differences of carbon emissions of animal husbandry in-depth, this study employs the Thiel index, kernel density analysis, and convergence analysis methods to systematically evaluate the sources and convergence of carbon emissions of animal husbandry. *Secondly*, this study divides the country into three areas: agricultural areas, intermingled agricultural–pastoral areas, and pastoral areas to perform a comparative analysis of the regional characteristics of carbon emissions of animal husbandry. *Thirdly*, the impact of livestock husbandry structure on carbon emissions of animal husbandry is explored using the econometric method to clarify the important sources of carbon emissions of animal husbandry.

The remainder of this study is organized as follows. Section Literature Review sufficiently gives relevant literature on carbon emissions of animal husbandry adequately. Section Methodology describes the model setting, variables selection, and data sources. Section Results and Analysis provides the empirical results and its relevant discussion. Finally, the research findings, policy implications, and further research directions are summarized.

## Literature Review

With the continuous development of animal husbandry, the resources invested in animal husbandry have increased. While promoting the economic development of animal husbandry, it has also caused certain negative impacts on the ecosystem and climate environment. This study collates the existing literature from two aspects: the estimation and source analysis of carbon emissions of animal husbandry and the influencing factors of carbon emissions of animal husbandry and to provide some inspiration for this study.

The contribution of livestock to greenhouse gas emissions is 15%, including about 37% of CH_4_ (22). For example, the carbon footprint of animal husbandry in China increased by 71% from 2005 to 2015 (6). The animal husbandry's carbon emissions mainly come from a large amount of excrement and urine carbon emissions produced by livestock and poultry farming, carbon dioxide and intestinal gas emissions produced by livestock and poultry breathing, carbon emissions generated by various wastes and pollutants in the livestock, and poultry farming process and other direct carbon emissions (23). However, in the process of livestock and poultry breeding, the indirect carbon emissions and environmental pollution caused by resource consumption cannot be ignored. Many scholars have found that cattle, sheep, and pigs are the key factors of greenhouse gas (GHG) emissions.

Income growth increases the demand for animal-based products rather than carbohydrates (24). The consumption of animal-based foods has increased rapidly over the decades (25). Increased meat consumption leads to increased production of livestock and poultry products, leading to greenhouse gas emissions from animal husbandry. Changing consumption habits should have a major impact on GHG emissions (26, 27). Meat consumption is significantly associated with physical health risks (28). Therefore, it is feasible to encourage consumers to eat less meat for consumption habits (9, 29, 30). Along these lines, it is necessary to change consumers' dietary behavior to reduce the impact of meat consumption on the environment (31–33). With the increasing population aging, the per capita meat consumption may decline; therefore, China's meat demand may be overestimated (34). With the rapid development of China's economy, meat consumption patterns and attitudes toward meat have changed (14). Pork is the most consumed meat globally, accounting for 45% of the total consumption (35). The GHG emission intensity of pork production is significantly lower than that of cattle (36). Therefore, changing consumption habits to reduce beef consumption and increase pork consumption will reduce carbon emissions.

As the second-largest source of carbon emissions, the environmental value of carbon emission reduction in agriculture cannot be ignored. Therefore, differentiated carbon reduction policies should be formulated according to regional differences. Recognizing the environmental problems caused by animal husbandry, the Chinese government has formulated many policies to promote fecal runoff control, fecal liquid-solid separation, biogas production, organic fertilizer, and environmental auditing of large livestock farms (37). At the same time, the government also establishes a carbon emission reduction market trading mechanism and compensation policy (38). With the continuous improvement of marketization, the appropriate collection of the carbon tax will also be conducive to low-carbon development (39). Due to the outbreak of the African Swine Fever in China in 2018, pork prices in China have risen sharply, and consumption of beef, mutton, and chicken has increased, which is advertised to greenhouse gas emissions of animal husbandry. Therefore, curbing pork prices has become an important task for the government (40). The outbreak of COVID-19 reduced social activities and carbon emission reduction (41). From January to July in 2020, the national catering income was 1,789.1 billion yuan, down 29.6% year on year, resulting in meat and cold chain loss. However, with the recovery of catering, meat consumption growth is also driven. Therefore, animal husbandry carbon emission management cannot be relaxed because of the epidemic.

The studies on the influencing factors of animal husbandry carbon emissions can be generally divided into two categories: macro influencing factors and micro influencing factors. The first is the analysis of macroscopic influencing factors. Among them, economic efficiency and production efficiency are the main factors to curb the carbon emissions of animal husbandry. For example, the impact of industrial structure, development level of animal husbandry, and education level of the labor force on carbon emissions vary from place to place. In contrast, the level of economic development, population and industrial scale, and level of animal husbandry have significant promoting effects on carbon emissions of animal husbandry (42). Dai et al. (36) used the Kaya identity and LMDI index to decompose the greenhouse gas emissions of China's pig industry. They found that the adjustment of agricultural structure, improvement of wealth, and population growth were important factors for increased carbon emissions. At the same time, the technological progress and structural change of animal husbandry were important reasons for carbon emission reduction. Rehman et al. (43) found that forestry production, rainfall, and temperature positively affected carbon emissions, while crop production, livestock production, energy use, and population growth had adverse effects on carbon dioxide emissions. Vigorously developing a circular economy and organically combining planting and animal husbandry can effectively reduce greenhouse gas emissions (16). The use of renewable biogas based on livestock waste and resource consumption based on a circular economy can play a mitigating role in climate change (44). Anaerobic digestion of animal manure and urban organic waste (MOW) for compressed biogas (CBG) production can effectively reduce greenhouse gas (GHG) emissions (45).

There are micro influencing factors as well, including household behavior, production mode, and environmental awareness (46, 47). Carbon emissions from animal husbandry are closely related to many factors, such as the quality of feed and intake level of livestock (48, 49). A feed with high-density fiber produces more methane, while home-grown feed has a small difference in the carbon footprint of livestock and poultry and can reduce methane emissions. Strengthening research on feed technology is conducive to reducing greenhouse gas emissions (50–52). In addition, the production model of animal husbandry also has a significant impact on greenhouse gas emissions (53–55). Sakamoto et al. (56) believe that the methane emission intensity under the intensive farming model is low. With the establishment of the social security system in pastoral areas, herders are more willing to participate in grassland ecological protection, which lays an important foundation for reducing carbon emissions and improving carbon sink capacity (57, 58). Carbon efficiency can be improved by introducing technology to change breeding management or ewe reproduction (59). The combined application of biogas BS and CF (chemical fertilizer) has the potential to reduce N_2_O emissions. Feed production and manure management are the main sources of GHG in pig production systems in China. Shifting to intensive pig production and improving feed crop planting and manure management systems will be key points to reducing GHG emissions from pig production systems (60).

To sum up, the existing research on carbon emissions of animal husbandry has achieved substantial outcomes in both theory and practice, but some gaps need to be further explored. Firstly, scholars simply compare the carbon emissions of animal husbandry both temporally and spatially, which makes it difficult to scientifically capture the distribution pattern of carbon emissions of animal husbandry (6, 22, 36). Li et al. (47), for example, reveal that carbon emissions from animal husbandry increased by 41% during the study period, and the increase in carbon emissions of animal husbandry was due to the increase in grazing intensity in the Qinghai-Tibet Plateau region, where cattle was the largest contributor of carbon emissions. Second, scholars primarily perform simple descriptive statistics on carbon emissions of animal husbandry, which can explain the regional differences in carbon emissions of animal husbandry but cannot effectively analyze the sources of differences and convergence (16). Zhang et al. (61) employ the SBM-Undesirable model to measure the carbon emission efficiency of the livestock industry in 13 prefecture-level cities (regions) in Heilongjiang province from 2005 to 2017 and verify that the overall carbon emission efficiency of the livestock industry in Heilongjiang Province shows a fluctuating upward trend. The carbon emission efficiency of the livestock industry has spatial and temporal differences. Finally, scholars pay more attention to regional carbon emissions of animal husbandry, while there are fewer investigations on the characteristics and influencing factors of carbon emissions of animal husbandry as a whole (17, 62, 63). Therefore, using the provincial panel data from 2000 to 2018, a systematic quantitative analysis of the spatial and temporal regional characteristics, dynamic characteristics, and convergence characteristics of livestock husbandry carbon emissions, as well as the impact of livestock structure on carbon emissions of animal husbandry was performed by employing the Thiel index, kernel density analysis, and convergence analysis methods.

## Methodology

### Emissions Factor Method

The methods for measuring carbon emissions of animal husbandry are relatively mature, mainly the IPCC emission factor method and the life cycle method (10, 60, 64). The life-cycle method requires the measurement of carbon emissions of animal husbandry from the whole life-cycle of livestock in six segments, including feed growing, feed processing, livestock feeding, gastrointestinal fermentation, manure fermentation, and livestock slaughter. Referring to Li et al. (47), this study employs the emission factor method to measure the carbon emissions of animal husbandry. The specific measurement of carbon emissions of animal husbandry is as follows.


(1) $$\begin{array}{r} E=\sum_{i=1}^{n}T_{i}E_{i}^{c} \end{array}$$

where *E* denotes the carbon emissions of animal husbandry. *i* denotes the livestock species. $E_{i}^{c}$ denotes the carbon emissions coefficient. *T*_*i*_ denotes the average rearing period. The average rearing cycle needs to be adjusted because different livestock species have different rearing cycles (65). It is assumed that *M*_*i*_ denotes the slaughter volume (year) and *S*_*it*_ denotes the year-end stocking volume in this study. *L*_*i*_ denotes the life cycle of the *i*_*th*_ species of livestock. This study assumes that the life cycle of pigs, rabbits, and poultry is <1 year, which are 200, 105, and 55 days, respectively, then the average rearing period is $T_{i}=L_{i}\times \frac{M_{i}}{365}$. For other animals such as cattle with a life cycle longer than 1 year, then the average rearing period is $\frac{S_{it}+S_{i\left(t-\;1\right)}}{2}$.

According to the IPCC 2007 fourth assessment report, each unit of methane is equivalent to 25 units of carbon dioxide. Each unit of nitrous oxide is equivalent to 298 units of carbon dioxide. The methane emissions coefficients of animal gastrointestinal fermentation and fecal fermentation are derived from IPCC's 2006 National Greenhouse Gas inventory guidelines. However, the nitrous oxide emissions coefficient of livestock manure fermentation in animal husbandry is calculated concerning the study of Zhuang and Li (1). The carbon emission coefficients are shown in Table 1.

**Table 1:** Carbon emissions coefficient of animal husbandry in China (unit: Kg/head/year).

**Species**	**CH**_**4**_		**N_**2**_O**	**CH**_**4**_ **→** **CO**_**2**_		**N_**2**_O → CO_**2**_**	***E* ^c^**
	**G1**	**G2**		**G1**	**G2**		
Pig	1	3.5	0.53	25	87.5	157.9	270.4
Rabbit	0.25	0.08	0.02	6.125	2	5.96	14.09
Poultry	0	0.02	0.02	0	0.5	5.96	6.46
Cow	68	16	1	1,700	400	298	2,398
Beef cattle	51.4	1.5	1.37	1,285	37.5	408.3	1,731
Horse	18	1.64	1.39	450	41	414.2	905.2
Donkey	10	0.9	1.39	250	22.5	414.2	686.7
Mule	10	0.9	1.39	250	22.5	414.2	686.7
Goat	5	0.17	0.33	125	4.25	98.34	227.6
Sheep	5	0.15	0.33	125	3.75	98.34	227.1
Camel	46	1.92	1.39	1,150	48	414.2	1,612

*G1 denotes the fermentation of intestines and stomach, G2 denotes the fermentation of feces*.

### Thiel Index Method

Referring to Theil and Uribe (66), this study employs the Thiel index method to investigate the spatial differences in carbon emissions of animal husbandry in China (66). The Thiel index was calculated as follows.


(2) $$\begin{array}{r} T=\frac{1}{n}\cdot \sum_{i=1}^{n}\frac{E_{i}}{\mu }ln\frac{E_{i}}{\mu } \end{array}$$

where n is the number of samples, i.e., 30 provincial administrative regions in China. *E*_*i*_ denotes the carbon emissions of animal husbandry in province *i*. μ denotes the average value of carbon emissions of animal husbandry in 30 provincial administrative areas in China.

### Kernel Density Method

This study applies kernel density analysis to investigate the dynamic evolution of carbon emissions in China's animal husbandry (67). Kernel density estimation is a nonparametric method that adopts a slipped peak function to fit the sample data and utilizes a continuous density curve to describe the distribution pattern of the variables. It does not involve setting up a functional form and can engrave the variables' variations with a continuous curve. This study sets the probability density of a group of random variables as *f*(*x*). Then, the expression of *f*(*x*) is as follows.


(3) $$\begin{array}{r} f\left(x\right)=\frac{1}{nh}\sum_{i=1}^{n}K\left(\frac{x-x_{i}}{h}\right) \end{array}$$

among them, *n* represents the number of observed samples, *h* represents the bandwidth, *x*_*i*_ represents the carbon emissions of animal husbandry in the *i* province and *K* (·) represents the kernel function, which is the weight function. Soentpiet (68) proposes that the Gaussian kernel function was superior to other kernel functions when the form of the function could not be determined. Therefore, the Gaussian kernel function was selected for research in this paper. The Gaussian kernel function is shown as follow:


(4) $$\begin{array}{r} K\left(x\right)=\frac{1}{\sqrt{2\pi }}e^{\left(-\frac{x^{2}}{2}\right)} \end{array}$$

### Convergence Analysis Method

Convergence analysis explains whether an index in different regions will shrink with time. If the index is reduced, which is convergence, otherwise it is divergence. The convergence analysis method is mainly divided into absolute convergence and conditional convergence. Absolute convergence is further divided into δ convergence and absolute β convergence. δ convergence can usually be expressed in terms of the coefficient of variation, i.e., a region in which an indicator is shrinking over time, then δ convergence is considered to be present. Referring to Zhuang and Li (1), we use the δ convergence method and σ convergence and absolute β convergence to verify the variance of carbon emissions in China's animal husbandry. The specific measurement is as follows.


(5) $$\begin{array}{r} CV=\frac{\delta }{\mu }=\frac{1}{\mu }\sqrt{\frac{1}{n-1}\cdot \sum_{i=1}^{n}{\left(E_{i}-\mu \right)}^{2}} \end{array}$$

where σ denotes standard deviation and μ for mean value. The absolute β converges as shown in Equation (6):


(6) $$\begin{array}{r} \frac{1}{t}ln\frac{E_{i,t}}{E_{i,1}}=\alpha +\beta lnE_{i,t}+\varepsilon_{i,t} \end{array}$$

where, *E*_*i*, 1_ represents carbon emissions of animal husbandry in the initial period of the *i* province. *E*_*i, t*_ represents carbon emissions of animal husbandry in the *t* period of the *i* province. β represents the convergence coefficient. If it is significantly negative, indicating absolute convergence. ε represents the random error term. Conditional convergence is mainly represented by conditional β convergence. The measurement of conditional β convergence formula is as follows:


(7) $$\begin{array}{r} lnE_{i,t}-lnE_{i,t-1}=\alpha +\beta {lnE_{i,t}}_{-1}+\varepsilon_{i,t} \end{array}$$

(8) $$\begin{array}{r} lnE_{i,t}=\alpha +\left(\beta +1\right){lnE_{i,t}}_{-1}+\varepsilon_{i,t} \end{array}$$

where β represents the conditional convergence coefficient. If it is significantly negative, it indicates that the variable has conditional convergence.

### Benchmark Regression Model Construction

In order to investigate the effect of livestock structure on carbon emissions from animal husbandry, the following economic model is constructed in this study Wang et al. (69).


(9) $$\begin{array}{r} AC_{i,t}=\beta_{0}+\beta_{1}Structure_{i,t}+\beta_{2}X_{i,t}+u_{i}+v_{t}+\varepsilon_{i,t} \end{array}$$

where *i*represents the provincial administrative area, and *t* represents the year. α and β represents the coefficient vector, respectively. *u* is the area fixed effect, and *v* is the time fixed effect. ε is the random disturbance term. The dependent variable is carbon emissions of animal husbandry (*AC*). The core explanatory variable is livestock structure. X is a group of control variables, including agricultural structure (*IND*), urbanization (*URB*), income level (*INC*), transportation accessibility (*POS*), and income gap (*ENG*).

### Variables Definition

#### Dependent Variable

Carbon emissions of animal husbandry (*AC*). The measurement of carbon emissions of animal husbandry is described in Section in Emissions Factor Method.

#### Core Explanatory Variable

Livestock structure (*STU*). Referring to Fu et al. (70), this study converts poultry, cattle, and sheep into pig equivalents and uses pigs to indicate the number of other livestock breeds. In this way, the share of poultry and pigs in all livestock breeds can be accounted for and used to indicate the structure of livestock breeds.

#### Control Variables

To control the influence of other factors on carbon emissions of animal husbandry, the following control variables are introduced, including five variables such as including agricultural structure (*IND*), urbanization (*URB*), income level (*INC*), transportation accessibility (*POS*), and income gap (*ENG*). Agricultural structure embodies changes in production and consumption structures, which have a significant impact on carbon emissions of animal husbandry. Therefore, referring to Yao et al. (17), the share of value-added of livestock in value-added of agriculture is used to measure the agricultural structure (*IND*). An increase in urbanization level drives economic development (71), which in turn leads to an increase in the residents' demand for livestock and poultry products. Following Wu et al. (72), the ratio of the permanent urban population to the total number of people is used to measure urbanization (*URB*). A change in income level is directly related to the demand for livestock and poultry products. Following Huo et al. (73), income level (*INC*) is introduced into the model as a control variable, which is expressed as annual per capita income. Transportation accessibility accelerates product distribution with important implications for the consumption of livestock and poultry products (69). This study uses road area per capita to measure transportation accessibility (*POS*). The income gap affects the marginal propensity to consume of the whole society, which in turn has an impact on livestock and poultry products consumption. Following Huimin and Dake (74), the income gap (*ENG*) is characterized by Engel's coefficient.

### Data Source

This study applies the relevant data of Chinese provincial administrations from 2000 to 2018 to test the effect of livestock structure on carbon emissions of animal husbandry, the spatial-temporal evolution, and convergence characteristics of carbon emissions of animal husbandry. Due to the unavailability of data, Tibet, Hong Kong, Macao, and Taiwan are not included in the analysis. The data for empirical analysis were derived from China rural statistical yearbook, China statistical yearbook, China statistical yearbook wind database, and prospective database^4^. Variable definitions are shown in Table 2.

**Table 2:** Variable definitions.

**Variable**	**Obs**	**Mean**	**Std. Dev**.	**Min**	**Max**
AC	570	12,109.06	8,790.986	413.58	45,345.33
STU	570	71.91384	23.68239	0.38	97.66
IND	570	87.8303	6.492473	63.55	99.68
URB	570	50.50621	15.02015	23.2	89.6
INC	570	7,078.021	5,109.673	1,374.16	30,374.73
POS	570	118,622.7	71,148.22	4,987	281,181.4
ENG	570	38.97044	8.003126	23.78	62.68

## Results And Analysis

### Analysis of the Measurement Results of Carbon Emissions of Animal Husbandry

According to Equation (1), the study calculates carbon emissions of animal husbandry in 30 provincial administrative areas in China. We further divide 30 provincial-level administrative areas into the pastoral, agro-pastoral, and agricultural areas to analyze the current characteristics of carbon emissions of animal husbandry in more detail (see Figure 2)^5^. Figure 2 depicts the overall trend of rising and then declining carbon emissions of animal husbandry. During the period from 2000 to 2006, carbon emissions of animal husbandry steadily increased and began to decline sharply after reaching a peak in 2006 (445,811.1 kilotons) and reached a minimum in 2009 (301,760.1 kilotons), and then finally increased slowly and showed an overall downward trend. The trend of carbon emissions of animal husbandry in the agro-pastoral interlocking areas, agricultural areas, and the whole country is consistent, and all of them achieved carbon peaking in 2006, which is also in line with the findings of Zhang and Wang (65). Zhang and Wang (65) suggest that China's carbon emissions from animal husbandry peaked in 2006. The overall variation of carbon emissions from animal husbandry shows a fluctuating and small increase, with the regional variation being the main source of the overall variation. Judging from the proportion of carbon emissions of animal husbandry in each area, the agricultural area has the largest proportion of carbon emissions with an overall decreasing trend, followed by the agro-pastoral area, with a small decreasing trend. On the contrary, the carbon emissions ratio of pastoral areas is the lowest, with a steady increase in a small way. One possible explanation is that livestock and poultry products are the main consumer goods for people, and their production is closely related to the consumer market. From the perspective of regional consumer distribution, China's densely populated areas are mainly distributed in agricultural and agro-pastoral areas. The main production positions of livestock and poultry products are consistent with consumer areas (17). During the study period, with the introduction of animal husbandry industry standards, the substandard livestock husbandry production in agricultural areas and agro-pastoral ecotone was suspended, resulting in a decline in carbon emissions in agricultural and agro-pastoral areas. However, there is a large area of grassland in pastoral areas (75). Herbivorous livestock husbandry has a large scale, which is relatively less affected by industry standards, so the carbon emissions of animal husbandry have increased.

**Figure 2:** Calculated results of carbon emissions of animal husbandry from 2000 to 2018 (unit: thousand tons).

### Analysis of the Temporal and Spatial Characteristics of Carbon Emissions of Animal Husbandry

In addition, to more intuitively depict the spatial differences of carbon emissions of animal husbandry, this study draws the spatial distribution map of carbon emissions of animal husbandry (see Figure 3) (76, 77). As can be seen from the spatial distribution map of carbon emissions of animal husbandry, the provinces with high carbon emissions of animal husbandry are gradually shrinking, and the carbon emissions of animal husbandry show regional heterogeneity (Figure 3). The provinces with the highest carbon emissions of animal husbandry in China in 2018 were Sichuan and Inner Mongolia.

**Figure 3:** Change and distribution of carbon emissions of animal husband.

Table 3 presents the temporal differences in carbon emissions of animal husbandry in China using the Thiel index to characterize each area. Table 3 reveals that the overall carbon emissions of animal husbandry showed a trend of rising and then declining with a maximum value of 0.2682 in 2009, indicating that the overall difference in carbon emissions of animal husbandry showed small fluctuations. In terms of spatial distribution characteristics, the Thiel index is the largest in agricultural areas, the second-largest in agro-pastoral interlacing areas, and the smallest in pastoral areas, which indicates the development of animal husbandry in agricultural areas is significantly different. In contrast, the development of the pastoral regions is less heterogeneous. The large difference in carbon emissions of animal husbandry in non-pastoralist areas may be mainly influenced by the degree of concentration of livestock and poultry farming. On the one hand, the consumer population is mainly concentrated in China's agricultural and agro-pastoral interlacing areas, thus causing significant demand for livestock and poultry products (31). However, the degree of concentration of consumer population in the agricultural areas and the agro-pastoral interlacing areas is highly variable, which leads to significant regional heterogeneity in livestock and poultry farming (78). On the other hand, influenced by natural conditions and environmental regulations, the heterogeneity of livestock and poultry farming in agricultural and agro-pastoral areas is more evident. Thus, the carbon emissions of animal husbandry show more significant differentiation (17).

**Table 3:** Theil index of carbon emissions of animal husbandry.

**Year**	**The total**	**Pastoral**	**Agro-pastoral**	**Agriculture**
	**area**	**area**	**area**	**area**
2000	0.2551	0.0235	0.2063	0.3075
2001	0.2515	0.0213	0.2082	0.3018
2002	0.2514	0.0211	0.2070	0.3024
2003	0.2489	0.0271	0.1939	0.3018
2004	0.2531	0.0397	0.1826	0.3089
2005	0.2571	0.0513	0.1807	0.3126
2006	0.2643	0.0593	0.1821	0.3207
2007	0.2638	0.0569	0.1700	0.3172
2008	0.2634	0.0550	0.1685	0.3028
2009	0.2682	0.0784	0.1674	0.2946
2010	0.2539	0.0878	0.1404	0.2828
2011	0.2463	0.0771	0.1209	0.2878
2012	0.2462	0.0680	0.1223	0.2919
2013	0.2447	0.0600	0.1200	0.2928
2014	0.2470	0.0583	0.1194	0.2972
2015	0.2545	0.0631	0.1195	0.3058
2016	0.2561	0.0611	0.1181	0.3080
2017	0.2554	0.0537	0.1208	0.3024
2018	0.2602	0.0511	0.1320	0.2987

The temporal trend shows that the Thiel index decreased for agricultural and mixed agro-pastoral areas while it increased for pastoral areas. More specifically, the Thiel's index for agricultural areas decreased from 0.3075 in 2000 to 0.2987 in 2018. Thiel's index for agro-pastoral areas decreased from 0.2063 in 2000 to 0.1320 in 2018, while the Thiel's index for pastoral areas increased from 0.0235 in 2000 to 0.0511 in 2018. The above results show that although the difference between agricultural and agro-pastoral areas is greater than that of pastoral areas, the degree of difference between agricultural and agro-pastoral areas is gradually decreasing, while the difference between pastoral areas is increasing. It is obvious that cattle and sheep farming are the main focus in terms of livestock breeds. Although the demand for beef and sheep meat in China is rising year by year, there are differences in the development of animal husbandry in Xinjiang, Qinghai, and Inner Mongolia, which leads to an increase in the differences in carbon emissions from animal husbandry (75).

### Analysis of the Dynamic Evolution Characteristics of Carbon Emissions of Animal Husbandry

Figure 4 reveals the results of estimating the dynamic effects of carbon emissions from livestock husbandry using the kernel density method. Specifically, from 2000 to 2018, China's livestock husbandry carbon emissions exhibited a single-peak characteristic, indicating that overall carbon emissions are homogenized. Regarding the height of the primary peak, China's livestock husbandry carbon emissions show a fluctuating change trend of first downward and then upward, which reached the highest value in 2010, indicating the differences of China's livestock husbandry carbon emissions among areas show fluctuating changes. In addition, the kernel density center shows a rightward and leftward shift characteristic, indicating that the carbon emissions of livestock husbandry in each area of China increase first and then decrease. From the trailing perspective, there is an evident phase of the right trailing phenomenon in livestock husbandry carbon emissions from 2000 to 2018, which experiences the evolution trend of “widening-convergence-widening”, indicating that there is a significant dynamic change of livestock husbandry carbon emissions (expanding and shrinking in each area).

**Figure 4:** Dynamic changes of carbon emissions of animal husbandry result. **(A)** The total area. **(B)** Pastoral areas. **(C)** Agro-pastoral areas. **(D)** Agricultural area.

In addition, the kernel density of carbon emissions from husbandry in pastoral areas shows different results. In terms of peak value, carbon emissions of animal husbandry from 2000 to 2018 also exhibit single-peak characteristics, indicating that carbon emissions are homogenized. From the height of the primary peak, the kernel density of carbon emissions of animal husbandry in pastoral areas showed a decreasing trend from 2000 to 2010. It then showed an increase afterward, which indicates that the differences in carbon emissions of animal husbandry in various areas show fluctuating changes from high to low. The distribution of kernel density center reveals that the kernel density center of carbon emissions of animal husbandry in pastoral areas shows a rightward shift characteristic from 2000 to 2005, after which the change of kernel density center is insignificant, suggesting that the carbon emissions of animal husbandry in each province and region increase and later decrease. The trailing phenomenon reveals that the right trailing phenomenon of the kernel density of carbon emissions of animal husbandry from 2000 to 2018 is not obvious, which indicates that the differences in carbon emissions of animal husbandry between pastoral areas are relatively low.

An unexpected result is that the kernel density of carbon emissions of animal husbandry in agricultural areas shows characteristics that are largely in line with those of the total area. From the peak value, the kernel density distribution of animal husbandry carbon emissions shows a single peak characteristic from 2000 to 2015 while showing a large and small peak characteristic in 2018, indicating that carbon emissions are mainly a unitary pattern. However, there is a possibility of multi-polarization. From the height of the primary peak, the change of the kernel density of carbon emissions of animal husbandry from 2000 to 2005 is low, rising to the highest point in 2010 and start falling in 2015, then rising again in 2018. This trend indicates that the difference in carbon emissions of animal husbandry in each area shows fluctuating changes. In addition, the kernel density of carbon emissions of animal husbandry shows a left-shifting characteristic, which indicates that the carbon emissions of animal husbandry in each area show a dynamic change characteristic of decline. From the trailing effect, the kernel density of carbon emissions of animal husbandry from 2000 to 2018 shows an apparent right trailing feature, indicating significant differences in animal husbandry carbon emissions in agricultural areas. These differences present the dynamic change characteristics of narrowing, expanding, and again narrowing.

### Analysis of Carbon Emissions of Animal Husbandry Convergence Result

Figure 5 reveals the convergence scenario of carbon emissions of animal husbandry in China using the coefficient of variation method. It can be observed that the coefficients of variation of carbon emissions of animal husbandry in pastoral, agro-pastoral, and agricultural areas, as well as in the total area, show a small trend of variation. Although the coefficients of variation of carbon emissions of animal husbandry in the total area and the agricultural area are higher, the changes are low, which indicates that there is no δ convergence of carbon emissions of animal husbandry in the total area and the agricultural area. The variation coefficients of carbon emissions of animal husbandry in pastoral and agro-pastoral areas are more significant. Among them, the coefficient of variation of carbon emissions of animal husbandry in pastoral areas changes from low to high with a maximum value in 2010 and then decreases slowly. The coefficient of variation of carbon emissions of animal husbandry in agro-pastoral areas shows a gradual downward trend overall. Still, there is a slow upward trend since 2016, which indicates that there is also no δ convergence in pastoral, and agro-pastoral areas.

**Figure 5:** δ convergence result.

Table 4 reports the estimation results for the absolute β convergence. Table 4 reveals that the β values of carbon emissions of animal husbandry are significant whether in the total area, pastoral area, agro-pastoral area, or in the agricultural area. Meanwhile, carbon emission levels are higher in pastoral areas than in agricultural areas, as well as there is a trend of convergence in performance levels across regions. However, β > 0 indicates that there is no absolute β convergence of carbon emissions of animal husbandry in each area. Moreover, the coefficient of β also indicates that the convergence is faster within pastoral areas, followed by agricultural areas, and slowest in agro-pastoral areas. In order to further facilitate the convergence and reduce the differences in carbon emissions among different regions, it is necessary to take certain policy measures to strengthen the exchange and communication between regions in terms of carbon reduction technology and management system arrangement so as better to promote the diffusion of advanced technology and management concepts. Table 5 reports estimation results of conditional β convergence, revealing that the (β+1) values of carbon emissions of animal husbandry are significant in total, pastoral, agro-pastoral, and agricultural areas. However, (β+1) > 0 indicates that there is no conditional β convergence of carbon emissions of animal husbandry in each area.

**Table 4:** Absolute β convergence result.

**Convergence**	**Total**	**Pastoral**	**Agro-pastoral**	**Agricultural**
	**area**	**area**	**area**	**area**
β	0.0625***	0.0910***	0.0174**	0.0620***
	(0.003)	(0.009)	(0.007)	(0.004)
α	−0.5654***	−0.8767***	−0.1447**	−0.5561***
	(0.029)	(0.093)	(0.067)	(0.033)
Ob.	570	57	114	399
N. of id	30	3	6	21

Standard errors in parentheses; ***p < 0.01, **p < 0.05.

**Table 5:** Conditional β convergence result.

**Convergence**	**(1)**	**(2)**	**(3)**	**(4)**
	**Total**	**Pastoral**	**Agro-pastoral**	**Agricultural**
	**area**	**area**	**area**	**area**
β+1	0.8869***	0.8572***	0.8024***	0.8962***
	(0.022)	(0.059)	(0.053)	(0.026)
α	1.0126***	1.4060**	1.8563***	0.9005***
	(0.200)	(0.579)	(0.492)	(0.235)
Observations	540	54	108	378
R-squared	0.760	0.807	0.698	0.763
Number of id	30	3	6	21

Standard errors in parentheses; ***p < 0.01, **p < 0.05.

### Analysis of Benchmark Regression Result

To validate the robustness of results, the regression results of the panel fixed effects (FE), random effects, and OLS models are also given (see Table 6). The regression results show that the structure of livestock restrains the increase of carbon emissions of animal husbandry, and the coefficient of livestock structure is significantly negative at a 1% confidence level. The reasons for this result are as follows. Firstly, the livestock structure reflects the proportion of poultry and pigs in animal husbandry. The carbon emissions coefficient of poultry and pigs is lower than that of ruminants, cattle, and sheep, so the higher the livestock structure, the lower the carbon emissions of animal husbandry (65). Second, with the rising income level in China, Chinese residents' consumption of beef and mutton has gradually increased. To enrich people's meat pots, the Chinese government encourages and supports the development of animal husbandry, especially the regulation and subsidies of pig breeding (60). Chen et al. (60) report that China's pig production system has moved toward having a positive impact on GHG emission reduction and that the pig industry still has considerable potential for GHG emission reduction. For example, the Chinese government has successively promulgated the national plan for the development of live pig production (2016–2020), the guiding opinions on accelerating the development of modern animal husbandry in the main grain-producing areas in the northeast (2017), and the opinions on stabilizing live pig production for transformation and upgrading (2019). The livestock structure has gradually improved, and the carbon emissions of livestock husbandry have shown a decreasing trend. Third, as China's aging population continues to rise, China's consumption of animal products should gradually decline according to the elderly's idea of less meat consumption to relieve the pressure on the development of animal husbandry and promote the high-quality development of animal husbandry.

**Table 6:** Benchmark regression result.

**Variables**	**(1)**	**(2)**	**(3)**	**(4)**	**(5)**	**(6)**
	**OLS**	**OLS**	**FE**	**FE**	**RE**	**RE**
Structure	−0.3621***	−0.6346***	−0.1381***	−0.1745***	−0.1427***	−0.1880***
	(0.073)	(0.042)	(0.046)	(0.041)	(0.046)	(0.042)
Industry		−2.0987***		−0.7963**		−0.7742**
		(0.402)		(0.348)		(0.364)
Urban		−0.9970***		−0.0231		−0.1910
		(0.143)		(0.125)		(0.130)
Income		−0.0141		−0.1408***		−0.1151***
		(0.053)		(0.031)		(0.033)
Postal		0.7156***		−0.0431		0.1287***
		(0.026)		(0.048)		(0.045)
Engel		−0.5158***		−0.2306***		−0.2470***
		(0.135)		(0.062)		(0.066)
Constant	10.5608***	18.8011***	9.6255***	15.9725***	9.6447***	14.4623***
	(0.306)	(1.805)	(0.194)	(1.503)	(0.260)	(1.550)
Observations	570	570	570	570	570	570
R-squared	0.042	0.769	0.016	0.249		
Number of id	30	30	30	30	30	30

Standard errors in parentheses; ***p < 0.01, **p < 0.05.

### Analysis of Robustness Test Result

This study performs robustness tests in two aspects. (1) Excluding idiosyncratic sample values. There are more idiosyncrasies between Chinese municipalities and other provincial-level administrative regions, so following Song et al. (79), this study excludes sample data from four municipalities (Beijing, Shanghai, Tianjin, and Chongqing) to re-estimate the empirical results (see columns 1 and 2 of Table 7). Second, the endogeneity test is executed. Referring to Wang et al. (69), the 2-lagged period of animal husbandry structure is selected as the instrumental variable. The empirical results are regressed again using the two-stage least square method (2SLS) (see columns 3 and 4 of Table 7). This study reveals that animal husbandry structure still significantly inhibits carbon emissions from animal husbandry, thus implying that the results of this study are robust.

**Table 7:** Robustness test result.

**Variables**	**(1)**	**(2)**	**(3)**	**(4)**
	**Excluding idiosyncratic sample values**	**Excluding idiosyncratic sample values**	**2SLS**	**2SLS**
Structure	−0.1563***	−0.1962***	−0.3976***	−0.7079***
	(0.044)	(0.039)	(0.080)	(0.049)
Industry		−0.9844***		−2.1575***
		(0.334)		(0.422)
Urban		−0.3316**		−0.9762***
		(0.131)		(0.153)
Income		−0.0353		−0.0072
		(0.035)		(0.055)
Postal		−0.0248		0.7336***
		(0.047)		(0.028)
Engel		−0.1903***		−0.4119***
		(0.063)		(0.140)
Constant	9.9553***	17.0562***	10.7049***	18.6558***
	(0.183)	(1.456)	(0.336)	(1.879)
Observations	494	494	540	540
R-squared	0.026	0.267	0.042	0.768
Number of id	26	26	30	30

Standard errors in parentheses; ***p < 0.01, **p < 0.05.

## Conclusions And Policy Implications

It is necessary to formulate effective emissions reduction policies to clarify the regional differences, dynamic evolution patterns, and structures of carbon emissions of China's animal husbandry. This study verifies the impact of livestock structure on carbon emissions of animal husbandry using panel data of provincial administrative regions in China from 2000 to 2018. Firstly, this study estimates the carbon emissions of animal husbandry in provincial administrative regions of China through the emission factor analysis method and then investigates the spatial and temporal evolution and convergence characteristics of carbon emissions of animal husbandry using kernel density estimation, Thiel's index method, and convergence analysis method. Further, this study examines the effect of livestock structure on carbon emissions of animal husbandry. Major findings include the following. There is a rising and then declining carbon emissions trend from animal husbandry. In terms of different regions, the share of carbon emissions of animal husbandry in agricultural areas is the largest with an overall declining trend; the share of carbon emissions of animal husbandry in intermingled agricultural and pastoral areas is the second largest with a slightly declining trend; the share of carbon emissions of animal husbandry in pastoral areas is the lowest, but shows a steady rise in a small range. In terms of spatial distribution, the differences between provinces/regions with high carbon emissions of animal husbandry gradually narrow and show significant spatial heterogeneity characteristics. Moreover, the carbon emissions of the animal husbandry industry did not pass the convergence test. Finally, livestock structure significantly inhibits carbon emissions of animal husbandry.

In order to reduce carbon emissions of animal husbandry through a reasonable livestock structure, some necessary policy implications should be performed.

1. Policymakers should strengthen the regulated development of animal husbandry and animal husbandry management to reduce carbon emissions of animal husbandry. For example, policymakers can establish a relevant leadership group in the livestock sector in each region and assign responsibility for the corresponding carbon emission reduction targets to individuals and posts to ensure the successful implementation of carbon emission reduction work. In line with the spatial heterogeneity of carbon emissions of animal husbandry, policymakers should adopt differentiated policies to ensure sufficient animal husbandry products while focusing on improving the quality of animal husbandry development and reducing carbon emissions.
2. Policymakers should further optimize the structure of livestock and poultry, raising the share of pigs and poultry in animal husbandry and reducing the share of cattle and sheep in animal husbandry. The culture of catering influences people's demand for livestock and poultry products, so optimizing the structure of livestock and poultry is more difficult. Policymaking should play the function of government and social organizations to change restaurant culture, progressively reduce the proportion of beef and sheep meat consumption, and reduce the carbon emissions of animal husbandry at the demand side.
3. Policymakers should strongly motivate livestock production enterprises to carry out research and develop low-carbon equipment actively and fully realize the transformation of technical achievements. Through government guidance, a low-carbon technology development system and application system for animal husbandry integrated with industry-university research is established as a way to reduce carbon emissions in animal husbandry.
4. Policymakers should strengthen international trade and international cooperation of animal husbandry products through worldwide coordination of animal husbandry product resource allocation to maximize the global husbandry development structure and reduce the overall carbon emissions of animal husbandry. Furthermore, policymakers can also introduce advanced technologies, equipment, and management practices to improve the carbon emission reduction capacity of animal husbandry in order to ensure the low-carbon sustainable development of China's animal husbandry with advanced international technologies.

Although this study analyzes the influence of animal husbandry on carbon emissions of animal husbandry, there are still some limitations because of the constraints of sample size and method selection. For example, when this study investigates the effect of livestock structure on carbon emissions of animal husbandry in a regional heterogeneity context, the empirical results are not desirable owing to the small sample size of the study after grouping. Therefore, future research can utilize analytical methods such as big data or the data at the prefecture level to carry out specific analyses of the above results to yield more accurate results. Moreover, industrial agglomeration, climatic conditions, and people's preference for meat may also be major factors influencing livestock structure and carbon emissions of animal husbandry. Therefore, the above perspectives can be used to diversely evaluate their significant impacts on carbon emissions of animal husbandry in the future.

## Data Availability Statement

The original contributions presented in the study are included in the article/supplementary material, further inquiries can be directed to the corresponding author/s.

## Author Contributions

RS: conceptualization, project administration, writing—review and editing, and writing—original draft. XY: writing—review and editing, software, and validation. GL: writing—review and editing and validation. MI: formal analysis, writing—original draft, writing—review and editing, validation, methodology, and data curation. XS: writing—review and editing, writing—original draft, conceptualization, methodology, funding acquisition, and supervision. All authors contributed to the article and approved the submitted version.

## Funding

The authors acknowledge financial support from the social Science Popularization and Application Research Project of Shandong Province (2020SKZZ31) and the Key Project of Xinjiang Social Science Foundation (19AZD008).

## Conflict of Interest

The authors declare that the research was conducted in the absence of any commercial or financial relationships that could be construed as a potential conflict of interest.

## Publisher's Note

All claims expressed in this article are solely those of the authors and do not necessarily represent those of their affiliated organizations, or those of the publisher, the editors and the reviewers. Any product that may be evaluated in this article, or claim that may be made by its manufacturer, is not guaranteed or endorsed by the publisher.

## Footnotes

^1^See more detail: https://www.fao.org/home/zh/

^2^See more detail: https://doi.org/10.1787/agr_outlook-2018-en

^3^At the Climate ambition summit on December 12, 2020, president Xi Jinping further outlines detailed arrangements for carbon peaking and carbon neutral targets, namely, “strive to achieve carbon peak by 2030 and carbon neutralization by 2060, China's carbon emissions will drop by more than 65% by 2030 compared to 2005, the share of non-fossil energy in primary energy consumption will reach about 25%”.

^4^See more detail: https://d.qianzhan.com/

^5^According to the classification criteria of China Animal Husbandry Association, we divide the study sample into three areas to explore the regional heterogeneity of livestock husbandry structure on livestock husbandry carbon emissions and the spatial and temporal distribution characteristics of livestock husbandry carbon emissions (pastoral, agro-pastoral and agricultural areas). Specifically, pastoral areas include Inner Mongolia, Qinghai and Xinjiang. The agro-pastoral areas include six provincial administrative areas, namely, Liaoning, Jilin, Heilongjiang, Sichuan, Gansu and Ningxia. Agricultural areas cover 21 provincial administrative areas, namely Beijing, Tianjin, Hebei, Shanxi, Shanghai, Jiangsu, Zhejiang, Anhui, Fujian, Jiangxi, Shandong, Henan, Hubei, Hunan, Guangdong, Guangxi, Hainan, Chongqing, Guizhou, Yunnan, and Shaanxi.
